The article "The Combination of Salidroside and Hedysari Radix Polysaccharide Inhibits Mitochondrial Damage and Apoptosis via the PKC/ERK Pathway" was published in 2022. Journal: Evid Based Complement Alternat Med.

# The Combination of Salidroside and Hedysari Radix Polysaccharide Inhibits Mitochondrial Damage and Apoptosis via the PKC/ERK Pathway

**DOI:** 10.1155/2022/9475703

**Published:** 2022-06-25

**Authors:** Sixia Yang, Linshuang Wang, Zeping Xie, Yi Zeng, Qiaowu Xiong, Tingting Pei, Dongfeng Wei, Weidong Cheng

**Affiliations:** ^1^School of Traditional Chinese Medicine, Southern Medical University, Guangzhou 510515, China; ^2^Institute of Basic Research in Clinical Medicine, China Academy of Chinese Medical Sciences, Beijing 100700, China

## Abstract

**Background:**

Beta-amyloid (A*β*) peptide is a widely recognized pathological marker of Alzheimer's disease (AD). Salidroside and Hedysari Radix polysaccharide (HRP) were extracted from Chinese herb medicine *Rhodiola rosea* L and *Hedysarum polybotrys* Hand-Mazz, respectively. The neuroprotective effects and mechanisms of the combination of salidroside and Hedysari Radix polysaccharide (CSH) against A*β*_25–35_ induced neurotoxicity remain unclear.

**Objective:**

This study aims to investigate the neuroprotective effects and pharmacological mechanisms of CSH on A*β*_25–35_-induced HT22 cells.

**Materials and Methods:**

HT22 cells were pretreated with various concentrations of salidroside or HRP for 24 h, followed by exposed to 20 *μ*m A*β*_25–35_ in the presence of salidroside or RHP for another 24 h. In a CSH protective assay, HT22 cells were pretreated with 40 *μ*m salidroside and 20 *μ*g/mL HRP for 24 h. The cell viability assay, cell morphology observation, determination of mitochondrial membrane potential (MMP), reactive oxygen species (ROS), and cell apoptosis rate were performed. The mRNA expression of protein kinase C-beta (PKC*β*), Bax, and Bcl-2 were measured by qRT-PCR. The protein expression levels of cleaved caspase-3, Cyt-C, PKC*β*, phospho-ERK1/2, Bax, and Bcl-2 were measured by Western blot.

**Results:**

CSH treatment increased cell viability, MMP, and decreased ROS generation in A*β*_25–35_-induced HT22 cells. PKC*β* and Bcl-2 mRNA expression were elevated by CSH while Bax was decreased. CSH increased the protein expression levels of PKC*β*, Bcl-2, and phospho-ERK1/2, and decreased those of Bax, Cyt-C, and cleaved caspase-3.

**Conclusions:**

CSH treatment have protective effects against A*β*_25–35_-induced cytotoxicity through decreasing ROS levels, increasing MMP, inhibiting early apoptosis, and regulating PKC/ERK pathway in HT22 cells. CSH may be a potential therapeutic agent for treating or preventing neurodegenerative diseases.

## 1. Introduction

Alzheimer's disease (AD) has an increasing number of patients, especially the elderly. Nowadays, AD affects approximately 40 million people and is expected to impact 135 million people by 2050 [1]. AD has imposed a heavy economic burden, which costs 0.65% of global gross domestic product (GDP) [2]. The clinical manifestations of AD include short-term memory difficulties, abnormal behavioral function (language expression, visuospatial processing, and execution), and personality changes. The neuropathologies of AD are characterized by amyloid-*β* (A*β*) deposition, neurofibrillary tangles (NFTs), which cause neuronal dysfunction, synapses loss in the hippocampus, and temporal cortex.

Neuronal apoptosis has been postulated as a possible explanation for the etiology of AD. Neurons displayed apoptotic characteristics, including apoptotic mitochondrial changes during AD progression [3]. Alteration in apoptosis-related factors may result in neurodegenerative diseases [4]. HT22 mouse hippocampal neuronal cells were usually used for underlying therapeutic mechanisms of neurodegenerative illness in place of primary neuronal cultures, and better mimic the pathological changes of AD neurons [5, 6]. Therefore, A*β*_25–35_-induced HT22 cells were used to explore the neuroprotective effects in this study [7].

Although there are many methods for treating AD [8], natural products are still an effective alternative treatment [9]. Salidroside extracted from the traditional Chinese medicine (TCM) *Rhodiola rosea* L. It has been shown that salidroside protects PC12 cells against the toxicity and apoptosis caused by A*β*_1–42_ through activating AKT and ERK1/2 pathways [10]. Hedysari Radix polysaccharide (HRP) is the major bioactive component derived from *Hedysarum polybotrys* Hand-Mazz. Studies have found that HRP attenuate A*β*-induced cell injury and improve the learning and memory in AD rats [11]. However, the neuroprotective effects and pharmacological mechanisms of the combination of salidroside and Hedysari Radix polysaccharide (CSH) against AD are unclear.

This study aimed to explore the neuroprotective effects and pharmacological mechanisms of CSH on A*β*_25–35_-induced HT22 cells. The cell viability assay, cell morphology observation, reactive oxygen species measurement, mitochondrial membrane potential detection, cell apoptosis detection, quantitative real-time PCR, and Western blot analysis were performed. The schematic diagram of experimental protocol is shown in Figure 1.

## 2. Materials and Methods

### 2.1. Materials

A*β*_25–35_ peptide was purchased from GL Biochem (Shanghai, China). Fetal bovine serum (FBS), penicillin/streptomycin, and trypsin were purchased from Gibco (Grand Island, USA). Salidroside (C10739039) was purchased from Macklin Biochemical (Shanghai, China). Hedysari Radix polysaccharide (wkq20041508) was purchased from Pythonbio (Guangzhou, China). Cell counting kit-8 (CCK-8) was purchased from Bimake (Houston, TX, USA). Hoechst 33342/PI double stain kit, JC-1 mitochondrial membrane potential fluorescent probe, and SDS-PAGE gels were purchased from Solarbio (Beijing, China). TRIzol® Reagen was purchased from Ambion (Austin, TX, USA). The Annexin V-FITC/PI double stain cell apoptosis detection kit was purchased from Keygen Biotech (Nanjing, China). The ROS assay kit was purchased from Jiancheng Bioengineering (Nanjing, China). The ChamQ SYBR® qPCR Master Mix kit was purchased from Affinity Biosciences (Cincinnati, OH, USA).

### 2.2. Cell Culture, A*β*_25–35_ Preparation, and Drug Treatment

HT22 mouse hippocampal neuronal cells were cultured in DMEM containing 10% FBS and 1% penicillin/streptomycin at 37°C in a humidity chamber with 5% (v/v) CO_2_. A*β*_25–35_ peptide was diluted to 1 mM with sterilized saline and then incubated at 4°C for 48 h to form aggregated A*β*_25–35_ before use [12]. In a cytotoxicity assay, HT22 cells were induced by different concentrations (5, 10, 20, 40, and 80 *μ*m) of A*β*_25–35_ for 24 h. In a drug protective assay, cells were pretreated with salidroside (10, 20, 40, 80, and 160 *μ*m) or RHP (10, 20, 40, 80, and 160 *μ*g/mL) for 24 h, respectively, followed by exposed to 20 *μ*m A*β*_25–35_ in the presence of salidroside or RHP for another 24 h. The cells in the control group were added with the same medium without A*β*_25–35_. In the CSH protective assay, cells were pretreated with 40 *μ*m salidroside and 20 *μ*g/mL HRP for 24 h, followed by exposed to 20 *μ*m A*β*_25–35_ in the presence of 40 *μ*m salidroside and 20 *μ*g/mL HRP for another 24 h.

### 2.3. Cell Viability Assay

This assay was conducted to demonstrate the neuroprotective effects of CSH against A*β*_25–35_-induced neurotoxicity. The viability of HT22 cells were evaluated by the CCK-8 assay. Briefly, after the treatment of A*β*_25–35_ or drug, the CCK-8 reagent was added to the cells, which were then incubated for 1.5 h at 37°C with 5% CO_2_ in dark conditions. The optical density (OD) was measured at an absorbance wavelength of 450 nm with a microplate reader (Multiskan FC, Thermo Scientific). Cell viability was normalized to the control.

### 2.4. Cell Morphology Observation

HT22 cells were seeded into 6-well plates. Cells in the CSH group were pretreated with CSH for 24 h, then induced by 20 *μ*m A*β*_25–35_ for 24 h. Cells in the A*β*_25–35_ group was treated with 20 *μ*m A*β*_25–35_ for 24 h. Cell morphology was observed under a light microscope (Olympus IX 53, Tokyo, Japan).

### 2.5. Measurement of ROS Generation

The reduction of oxidative stresses could reduce the onset of AD [13]. HT22 cells were seeded into 6-well plates and cultured as previously described. Cells were incubated at 37°C with 10 *μ*m DCFHDA for 30 min and washed 3 times. The level of ROS was detected by a fluorescence microscope (Olympus IX 53, Tokyo, Japan).

### 2.6. Determination of Mitochondrial Membrane Potential (MMP)

The decreased MMP is a characteristic in the early stage of cell apoptosis [14]. The A*β*‐mediated cytotoxicity and CSH intervention on MMP in HT22 cells were evaluated by JC-1 fluorescence. HT22 cells were cultured as previously described and stained with 10 *μ*g/mL JC-1 for 20 min at 37°C, after washed 3 times, a fluorescence microscope was used to observe the changes of MMP. With a typical negative membrane potential, JC-1 dye diffused into cells and entered mitochondria. The dye was subsequently collected in healthy mitochondria and fluoresces red. JC-1 remained distributed in the cell as a monomer and fluoresced green if MMP was disturbed.

### 2.7. Cell Apoptotic Morphological Assay

HT22 cells were cultured as previously described. Hoechst 33342 staining solution was made in accordance with the manufacturer's specified methodology, and 5 *μ*L Hoechst 33342 was added to 1 mL staining buffer and mixed well. 500 *μ*L Hoechst 33342 was incubated and protected from light. Cell apoptotic morphology was observed by a fluorescence microscope.

### 2.8. Detection of the Cell Apoptosis Rate

Neuronal cell injury and loss contribute to A*β*-induced apoptosis [15]. Therefore, cellular apoptosis was analyzed to confirm that CSH had a neuroprotective effect to antagonize A*β* neurotoxicity. HT22 cells were cultured as previously described and seeded in 6-well plates. Cells were harvested and resuspended in 100 *μ*L of binding buffer. Samples were incubated with 5 *μ*L Annexin-V-FITC and 5 *μ*L PI for 15 min at room temperature. 400 *μ*L of binding buffer was added, gently mixed. Samples were analyzed with flow cytometry (Beckman Coulter Cytoflex, USA).

### 2.9. Quantitative Real-Time PCR (qRT-PCR)

Total RNA was extracted using Trizol reagent according to the manufacturer's instructions. Total RNA was reverse transcribed to cDNA and amplified and analyzed using the ChamQ SYBR® qPCR Master Mix kit and a LightCycler96 PCR instrument (Roche, Mannheim, Germany). The mRNA expression of protein kinase C-beta (PKC*β*), Bcl-2, and Bax were analyzed using the 2^−ΔΔCt^ method and *β*-actin was set as internal reference. The primer sequences used are shown in Table 1.

### 2.10. Western Blot Analysis

To detect the expression levels of apoptosis-related proteins of HT22 cells, Western blot was performed. HT22 cells were collected and total cell protein was extracted from each group. After being quantified and denatured, electrophoresis was performed in a 12% polyacrylamide gel. 20 *μ*g total protein per sample of each group was added, after electrophoresis, transferring to the membrane. The membranes were blocked with 5% skim milk for 2 h and incubated with primary antibodies anti-Bcl-2 (lot 11o9905, Affinity Biosciences, Cincinnati, OH, USA), anti-Bax (Affinity, lot 44q6915), anti-PKC*β* (Affinity, lot 69q9084), anti-Cyt-C (Affinity, lot 73c2522), anti-cleaved caspase-3 (Affinity, lot 15z0096), anti-phospho-Erk1/2 (Cell Signaling Technology, lot 24, Boston, USA), anti-ERK1/2 (Servicebio, lot LS193349, Wuhan, China), and anti-*β*-actin (Affinity, lot: 7) overnight at 4°C. The membranes were washed 3 times and incubated with secondary antibody HRP-goat anti-rabbit IgG (Affinity, lot 20000135) for 1 h. After washing 3 times, ECL reagents (Vazyme, Nanjing, China) were added for chemiluminescent imaging. The protein bands were quantitatively analyzed by an ImageJ software.

### 2.11. Statistical Analysis

All statistical analyses were performed by SPSS 24.0. Results are expressed as mean ± standard deviation (SD). Comparisons among groups were analyzed using one-way analysis of variance (ANOVA) with the Tukey's posthoc multiple comparisons test. *P* < 0.05 was considered statistically significant.

## 3. Results

### 3.1. CSH Attenuated A*β*_25–35_-Induced Cytotoxicity in HT22 Cells

HT22 cells were exposed to different concentrations of A*β*_25–35_ for 24 h and 5–80 *μ*m of A*β*_25–35_-induced significant decrease of cell survival in a dose-dependent manner (*P* < 0.01) (Figure 2(a)). 20 *μ*m A*β*_25–35_ was used to induce cell injury in subsequent experiments. 40–160 *μ*m of salidroside significantly increased cell survival (*P* < 0.01) (Figure 2(b)). 20–160 *μ*g/mL of HRP significantly increased cell survival (*P* < 0.01). There were no significant differences in cell viability between 20–160 *μ*g/mL groups (*P* > 0.05) (Figure 2(c)). 40 *μ*m salidroside and 20 *μ*g/mL HRP were combined to against A*β*_25–35_-induced cell toxicity in subsequent experiments. CSH treatment significantly increased cell viability compared with the A*β*_25–35_ group (*P* < 0.01) (Figure 2(d)). The cell viability of CSH treatment was higher than that of 40 *μ*m salidroside treatment or 20 *μ*g/mL HRP treatment (*P* < 0.05). The results indicated that CSH attenuate A*β*_25–35_-induced cytotoxicity in HT22 cells.

### 3.2. CSH Protected Cell Morphology Damage

The cells were spindle-like and grew adherently, displaying some protrusions in the control group. The shrank and round cells and small cytoplasm protrusions on the cell surface were observed in the A*β*_25–35_ group. Compared with the A*β*_25–35_ group, the number of shrunk cells and cell gaps were markedly decreased in the CSH group, while adherent cells increased (Figure 2(e)). The results suggested that CSH protects A*β*_25–35_-induced cell morphology damage.

### 3.3. CSH Decreased ROS Production and Inhibited Cell Early Apoptosis

ROS production was increased in the A*β*_25–35_ group compared to the control group (*P* < 0.01). The levels of ROS were decreased after CSH treatment (Figures 3(a) and 3(b)). These results suggested that CSH could significantly protect HT22 cells from oxidative damage. The cell apoptotic morphology of HT22 cells identified by Hoechst 33342 staining are shown in Figure 3(c). The control group showed light blue staining. Compared to the control group, cells in the A*β*_25–35_ group showed shrinking nuclei and bright blue staining (*P* < 0.01). Compared to the A*β*_25–35_ group, bright blue cells decreased in the CSH group (*P* < 0.01). As shown in Figure 3(d), the apoptotic rate was analyzed by flow cytometry. The apoptosis rate was the sum of early and late apoptosis. Compared to the A*β*_25–35_ group, the early apoptosis rate was significantly decreased in the CSH group (*P* < 0.01) (Figure 3(e)). There were no significant differences in the late apoptosis rate between the CSH and A*β*_25–35_ groups. The percentage of apoptotic cells was scored and depicted graphically as shown in Figure 3(f). The results suggested that CSH can inhibit early apoptosis in A*β*_25–35_-induced HT22 cells.

### 3.4. CSH Increased Mitochondrial Membrane Potential (MMP)

As shown in Figure 4, JC-1 staining showed bright red fluorescence and weak green fluorescence in the control group. Cells in the A*β*_25–35_ group revealed a decrease in red fluorescence and a rise in green fluorescence, indicating a significant reduction of MMP (*P* < 0.01). CSH treatment inhibited MMP dissipation, which led to enhanced red fluorescence and decreased green fluorescence (*P* < 0.05). The results showed that the mitochondrial function of HT22 cells was significantly damaged by A*β*_25–35_ but restored by CSH. CSH inhibited A*β*_25–35_-induced apoptosis and exert a protective effect via maintaining high MMP.

### 3.5. CSH Regulated the mRNA Levels of PKC*β*, Bcl-2, and Bax

The mRNA levels of PKC*β*, Bcl-2, and Bax in HT22 cells were determined by a qRT-PCR assay. Compared with the control group, the Bax mRNA level was increased in the A*β*_25–35_ group, but decreased in the CSH group (*P* < 0.05). In the A*β*_25–35_ group, PKC*β* and Bcl-2 mRNA levels were decreased while they were higher in the CSH group (*P* < 0.05) (Figure 5(a)). These results indicated that CSH can inhibit apoptosis primarily through the intrinsic-apoptotic pathway in A*β*_25–35_-induced HT22 cells.

### 3.6. CSH Regulated Apoptosis-Related Proteins

The protein expression levels of PKC*β*, Bcl-2, Bax, Cyt-C, cleaved caspase-3, and phospho-ERK1/2 in HT22 cells were measured by Western blot. Compared with the control group, the protein expression levels of Bax, Cyt-C, and cleaved caspase-3 were increased in the A*β*_25–35_ group, while the protein expression levels of PKC*β*, Bcl-2, and phospho-ERK1/2 were decreased. Compared with the A*β*_25–35_ group, CSH treatment decreased the protein expression levels of Bax, Cyt-C, and cleaved caspase-3, and increased that of PKC*β*, Bcl-2, and phospho-ERK1/2 (Figure 5(b)).

## 4. Discussion

AD is mediated by multiple factors, with many theories of pathogenesis remaining unconfirmed [16]. Formed by aggregation of A*β* monomer and hyperphosphorylation of microtubule-associated protein Tau (p-Tau), A*β* plaques and neurofibrillary tangles (NFTs) were considered to be critical biomarkers in AD brains [17]. Apoptosis is a crucial point in A*β*-induced cytotoxicity, which includes promoting mitochondrial division, increasing intracellular ROS levels, and disrupting MMP [18]. Thus, the alleviation of A*β*-induced neuronal apoptosis seems to be a potentially curative treatment for AD [19]. This study showed that CSH decreased the A*β*_25–35_-induced early apoptosis rate in HT22 cells.

Deeply integrating theory and practice, TCM has shown promising efficacy in miscellaneous disorders for over 2,000 years [20], which has opened up new avenues to discover effective drugs and compounds for neurodegeneration, certainly including AD [21–23]. Salidroside, the main active ingredient in *Rhodiola rosea* L, was thought to help with mental and behavioral diseases when treated before the experimental injury [24]. Previous studies showed that salidroside contributed to relieving oxidative damage, decreasing TNF-*α*, IL-6 expression, and reducing hippocampus neuronal apoptotic rates in the AD mice model [25]. Salidroside had protective effects and alleviated PC12 cells damage induced by A*β*_1–40_ through the NAMPT signaling pathway [26]. Salidroside decreased the deposition of A*β*, and attenuated A*β*-mediated neurotoxicity by upregulating the PI3K/Akt/mTOR pathway in APP/PS1 mice [27, 28].

In TCM theory, herb processing significantly affects the medicinal property. *Hedysarum polybotrys* was the processed product of *Astragalus.* They have similar chemical constituents and both contain various polysaccharides. However, the total polysaccharide content of *Hedysarum polybotrys* was more than *Astragalus*. It was perhaps the reason for their differential pharmacological effects [29]. Recent studies have shown that RHP and Astragalus polysaccharides (APS) have anti-senescence effects. The mechanism might be the antioxidant capacity and attenuation of lipid peroxidation [30]. By maintaining physiological functions, RHP and APS could inhibit apoptosis of brain cells. Moreover, at the same dose, RHP showed a more substantial effect than APS on protecting neurite integrity, relieving the brain tissue lesions, and improving neurodegenerative disease [31]. HRP protected PC12 cells induced by A*β*_25–35_ via regulating the mitochondrial apoptotic pathway. In addition, RHP therapeutic properties targeting neuroblastoma cells apoptosis induced by A*β*_25–35_ have been confirmed by in vitro experiments [11].

Previous studies have demonstrated that elevated ROS can lead to cell death and dementia [32, 33]. ROS-induced lipid peroxidation can damage phospholipids and mediate proinflammatory change [34]. A*β*_1–42_ peptide abnormal production is associated with increased oxidative stress and an overabundance of inflammatory ROS, which ultimately leads to neuronal injury and death [35, 36]. Furthermore, high amounts of ROS promote the dissipation of MMP. Overloading intracellular Ca^2+^ caused mitochondrial depolarization, exacerbating oxidative stress-induced cell apoptosis [37]. Previous studies suggested that salidroside could inhibit the intracellular ROS level in PC12 cells, the A*β*_1–40_-induced AD rat model, and ultimately suppress cell apoptosis. However, the above studies did not focus on A*β*_25–35_-induced HT22 cells. In this study, higher ROS levels induced by A*β*_25–35_ were reduced by CSH treatment. Our findings demonstrated the antiapoptotic effect of CSH. These results were consistent with the apoptotic effects of salidroside in other disease models. A putative schematic model of pharmacological mechanisms of CSH inhibiting A*β*_25–35_-induced mitochondrial damage and apoptosis of HT22 cells is shown in Figure 6.

Neuronal loss and apoptosis were considered major mechanisms of cell death, which had an important implication on neurodegenerative diseases, notably AD [38, 39]. Apoptosis usually shows typical morphological features, chromatin condensation, such as nuclei shrinkage, nuclei fragmentation, and apoptosis body formation [40]. Both Bax and Bcl-2 are pivotal regulators in the intrinsic apoptosis pathway [41]. Bax could influence mitochondria-mediated cell death by three mechanisms. The first is to cleave Bax by cysteine protease [42]. The second was aided by an increased Bax/Bcl-2 ratio. The mitochondrial apoptotic pathway is driven by inhibitory interaction between Bax and Bcl-2 family [43]. The third way is related to translocated Bax to mitochondria so that mitochondrial permeability could be enhanced before apoptosis.

Similar to Bax, Bcl-2 regulates cell apoptosis via its activation in mitochondria and regulates the beginning of apoptosis [44]. Recent research showed that this antiapoptosis function was associated with the regulation of intracellular Ca^2+^ signaling. Aberrant Ca^2+^ signaling resulted in the dysregulated Bcl-2-Ca^2+^ signaling axis, ultimately accelerating AD pathology [45]. Ca^2+^ dysregulation and activated p38K caused increased ROS and decreased Bcl-2 levels in AD patients, leading to apoptosis [46]. In the present study, the mRNA and protein levels of Bax and Bcl-2 after CSH treatment were used as an assessment to detect A*β*_25–35_-induced HT22 cells apoptosis. CSH significantly decreased the protein expression and mRNA levels of Bcl-2 while increased that of Bcl-2 in A*β*_25–35_-induced HT22 cells.

PKC*β* belongs to the kinase C family and can negatively regulate the mitochondrial energy. Contributing significantly to cell proliferation, differentiation, and apoptosis, PKC*β* attenuated mitochondrial energy and reduced autophagy. The process was governed by multiple cell signaling pathways and diverse functions, including apoptosis induction, B-cell activation, and endothelial cell proliferation [47, 48]. Previous studies showed that PKC*β* could regulate neuronal function, which is associated with anxiety-related stress and contributes to conflict behaviors [49]. The precise molecular mechanisms underlying PKC*β*-mediated AD development remain obscure. Low expressions of PKC*β* was likely an underlying etiology of AD, potentially involving Fc*γ*R-mediated phagocytosis and the MAPK pathway [50].

ERK1/2 can regulate long-term neuronal plasticity and survival [51]. ERK1/2 expression can also be influenced by PKC*β* protein, protecting cells from A*β*-induced apoptosis. ERK1/2 has the potential to act as the target of Ca^2+^ signaling and was involved in granulosa cell apoptosis [52]. As a diagnostic marker, ERK1/2 displayed elevation in AD patients compared to healthy control, although it happens later than accumulated *t*-Tau and *p*-Tau [53]. In vitro and in vivo results proved that the ERK1/2 pathway would be activated by excitotoxic injury, exerting protective actions against damage, and neural loss [54]. The activation of the ERK1/2 induced cortical neuron apoptosis [55], and caused multiple changes of functional plastic in neuronal cells [56]. Both in clinical cases and AD mouse models, activated p38 MAPK has been observed in early-AD brain [57]. In this study, CSH treatment improved PKC*β* and phospho-ERK1/2 levels in mRNA and protein expression, which further confirmed the antiapoptotic effects of CSH.

However, several limitations still exist in this study. Cells were cultured in a simulated internal environment, which is still different from the in vivo environment of AD patients. In the future, the neuroprotective effects and pharmacological mechanisms of CSH treatment will be further investigated in AD animal models. It is difficult to find out the direct targets of CSH. Thus, the further studies may be necessary to clarify this.

## 5. Conclusion

In conclusion, the present study indicate that CSH treatment have protective effects against A*β*_25–35_-induced cytotoxicity in HT22 cells. CSH treatment increased cell viability through decreasing ROS levels, increasing MMP, inhibiting early apoptosis, and regulating the PKC/ERK pathway. The results of our study suggest that CSH may be a potential therapeutic agent for treating or preventing neurodegenerative diseases.

## Figures and Tables

**Figure 1:** Schematic diagram of experimental protocol.

**Figure 2:** Cell viability analysis and cell morphology observation of HT22 cells. (a) Different concentrations of A*β*_25–35_ on cell viability. Different concentrations of salidroside (b) RHP (c) and CSH (the combination of 40 *μ*m salidroside and 20 *μ*g/mL HRP) (d) on cell viability in A*β*_25–35_-induced HT22 cells. (e) The cell morphology of HT22 cells under a light microscope. Scale bar = 50 *μ*m ^*∗∗*^*P* < 0.01.

**Figure 3:** Effects of CSH on ROS levels and apoptosis in A*β*_25–35_-induced HT22 cells. (a) ROS generation were stained with DCFHDA, scale bar = 50 *μ*m. (b) Quantitative analysis of ROS generation. (c) Morphological apoptosis was determined by staining with Hoechst 33342, scale bar = 100 *μ*m. (d) Flow cytometric analysis of HT22 cells. (e) Quantitative analysis of the early apoptosis rate. (f) Quantitative analysis of the apoptosis rate. The apoptosis rate was quantified by sum of the early and late apoptosis rate. ^*∗∗*^*P* < 0.01.

**Figure 4:** Mitochondrial membrane potential in HT22 cells. The high-intensity red fluorescence indicates higher membrane potential, while the high-intensity green fluorescence indicates lower membrane potential. Scale bar = 50 *μ*m ^*∗∗*^*P* < 0.01.

**Figure 5:** Effects of CSH on markers of apoptosis in HT22 cells. (a) Relative mRNA levels of PKC*β*, Bcl-2, and Bax. (b) Representative Western blot results and quantitative analysis of PKC*β*, Bcl-2, Bax, Cyt-C, cleaved caspase-3, and phospho-ERK1/2 (p-ERK1/2) ^*∗*^*P* < 0.05, ^*∗∗*^*P* < 0.01.

**Figure 6:** A putative schematic model of pharmacological mechanisms of CSH increasing cell viability in A*β*_25–35_-induced HT22 cells. CSH inhibited apoptosis through regulating the PKC/ERK pathway and markers of apoptosis (cleaved caspase-3, Cyt-C, and Bax).

**Table 1:** Gene primer sequence used for qRT-PCR.

Gene	Forward primer (5′–3′)	Reverse primer (5′–3′)
PKC*β*	CAAGTCTGCTGCTTTGTTGTAC	TCTTAAACTTGTGTTTGCTCCG
Bcl-2	TGACTTCTCTCGTCGCTACCGT	CCTGAAGAGTTCCTCCACCACC
Bax	CCTTTTTGCTACAGGGTTTCAT	TATTGCTGTCCAGTTCATCTCCA
*β*-actin	CTACCTCATGAAGATCCTGACC	CACAGCTTCTCTTTGATGTCAC

## Data Availability

The data of this study are available from the corresponding author upon request.
